RETRACTED

# An optimal method for melanoma detection from dermoscopy images using reinforcement learning and support vector machine optimized by enhanced fish migration optimization algorithm

**DOI:** 10.1016/j.heliyon.2023.e21118

**Published:** 2023-10-17

**Authors:** Qianqian Liu, Hiroto Kawashima, Asad Rezaei sofla

**Affiliations:** a Laboratory of Microbiology and Immunology, Graduate School of Pharmaceutical Sciences, Chiba University, Chiba 260-8675, Japan; b University of Tehran, Tehran, Iran; c College of Technical Engineering, The Islamic University, Najaf, Iraq

**Keywords:** Melanoma detection, Feature selection, Reinforcement learning, Enhanced fish migration optimizer (EFMO), Feature extraction, Support vector machine

## Abstract

Early detection of melanoma is crucial in preventing death from this fatal skin cancer. Therefore, it would be valuable to develop a method that facilitates this process. The diagnosis of melanoma typically involves an invasive form of testing called a biopsy, as well as non-invasive intelligent approaches to diagnosis. In the present study a recent research, a novel approach has been developed for the optimal detection of melanoma cancer. The method uses reinforcement learning for segmenting the skin regions, followed by the extraction and selection of useful features using the Enhanced Fish Migration Optimizer (EFMO) algorithm. The outcomes get categorized on the basis of an optimized SVM on the basis of the EFMO algorithm. The recommended approach has been certified by applying it to the SIIM-ISIC dataset of Melanoma and comparing it with 12 other approaches. Simulations illustrated that the proposed method delivered the finest values compared to the others.

## 1 Introduction

### 1.1 Background

Skin cancer is a serious condition that can result in significant disability and high treatment costs. Melanoma has been considered the most unusual and dangerous kind of cancer in skin [1]. The goal of the current investigation is to study the epidemiology of skin cancer in Iran and the factors affecting it. According to statistical information from 2023, cancer of skin has been counted as the most typical kind of cancer worldwide, where numerous instances of non-melanoma cancer of skin occur yearly in the globe that its number is approximately 2 or 3 million, making it the most prevalent kind of cancer [2] (see Table 3).

It is important to note that not all skin cancers are melanomas, and the epidemiology and prevalence of different types of skin cancer may vary [3]. Therefore, skin cancer, including melanoma, is a significant public health issue that requires continued attention and research. Understanding the epidemiology and risk factors associated with skin cancer can help inform prevention and early detection efforts, which can improve outcomes for those affected by this disease [4]. If cancer is detected in the early stages, it will provide a significant impact on the definitive cure for this complication.

RETRACTED

Diagnosing melanoma in its initial phases can significantly decrease the potential of demise. However, early diagnosis can be challenging, even for specialists. Therefore, it is essential to provide efficient and effective ways of diagnosing melanoma in the initial phases [5]. If melanoma is detected early, more than 90 % of patients can be cured. However, only experienced physicians using appropriate tools and histological reports can diagnose malignancy promptly [6].

In addition to surgical procedures, several non-invasive methods are being tested to detect melanoma. These methods include digital photography, multispectral imaging systems, and dermoscopy. Novel approaches, such as Non-Invasive Diagnostic Assessment Tools, are also being developed in labs [7,8]. These approaches aim to enhance the efficacy and accuracy of detecting melanoma, particularly in its early stages.

Every one of the ground-breaking approaches possesses distinctive merits and demerits. practically, the finest approach has been chosen in accordance with the accuracy and efficacy as opposed to price considerations and comfort of usage, although, they are not the only variables of choice. The nature of the images that are used has a lot of weight, the size of the classes for example.

Dermatoscopic images are commonly used for diagnosing melanoma [8]. Early diagnosis of skin cancer is crucial, making it valuable to provide efficient techniques for detecting it in its early stages [9]. Recently, the usage of deep learning for diagnosing skin cancers has been increasing significantly.

The widespread adoption of new technologies in various fields, including medical applications, has led to the accumulation of large volumes of data. While this data can provide valuable insights for improving patient diagnosis and treatment methods, processing it is possible to be a time-consuming and challenging procedure [10].

### 1.2 Related works

Medical image processing is a widely-used application in healthcare analytics. There are several different techniques that were introduced in this field [11,12]. For example, Toğaçar et al. [13] detected malignant skin lesions intelligently with the help of the speaking neural network, auto encoder, and MobileNetV2. Melanomas are a kind of cancerous skin growth that gets developed through the pigment-generating cells, which have been named melanocytes. These growths can appear as multiple malignant lesions on the skin, typically showing up as dark, irregularly-shaped spots or moles. If left untreated, melanomas can can threaten life and spread to various organs. Therefore, prompt cure and timely diagnosis are crucial for managing this condition [14]. To diagnose melanoma, they used the CNN (Convolutiona Neural Network) technique. For evaluating the efficiency of the proposed artificial intelligence way, they used a cancer data set called ISIC, which contains 1800 images of malignant skin cancer [15]. The results showed that the accuracy of skin lesion detection by the neural network was 95.3 %. The results showed the high capability of artificial intelligence in diagnosing skin cancer.

RETRACTED

Kumar et al. [16] utilized the DE-ANN technique through C-Means fuzzy clustering to classify skin cancer. Early detection of skin lesions can help treat skin cancer. One method of identifying skin tumors is medical imaging. In the present case, they tried to help diagnose skin tumors by presenting a new method. They used fuzzy C-means clustering to classify skin lesions to diagnose disease. To achieve better results, they used the presented technique on skin tumor image datasets including HAM10000 and PH^2^. The results showed the suggested procedure acts more properly compared to other approaches to diagnosing malignant skin lesions. The classification results showed that the fuzzy method can detect about 97.4 % of skin tumor tumors.

Li et al. [17] distinguished malignant skin tumors using optimization techniques. Since skin cancer is very deadly among skin illnesses, early diagnosis of the disease contributes significantly to the medical community to treat the disease. Because of the significance of this issue, in the present research, they used the optimization way to enhance the recognition of lesions in skin. The optimization technique identifies the disease

in four steps, which include contrast, segmentation, extraction, and classification of the skin lesion image. The results indicated the fluid search optimization technique was able to make the best diagnosis for malignant skin lesions. The reason for this superiority was the high convergence speed in optimizing the detection steps and increasing the detection accuracy.

Astorino et al. [18] described an implementation of a MIL (Multiple Instance Learning) strategies for identification of melanoma, which was utilized to distinguish between negative and positive series of objects. Because an image was categorized based on some of its subdivisions, categorization of image is a suitable application for the paradigm of Multiple Instance Learning. The MIL algorithm outperforms typical classification algorithms regarding accuracy and sensitivity, with outcomes such as 92.50 % accuracy, 97.50 % sensitivity, and 87.50 % specificity. This shows that a MIL method might serve as the foundation for more complex tools that clinicians can utilize to diagnose melanoma.

RETRACTED

Zumpano et al. [19] presented a method using the paradigms of MIL for categorizing X-ray pictures of pneumonia into 3 categories: radiographic of healthy individuals, radiographic of individuals, who are diagnosed to have bacterial pneumonia, and radiographic of individuals with biological pneumonia. The suggested methods that have been quite quick in reality, look capable, particularly because no preprocessing strategy was applied.

Hasan et al. [20] identified malignant skin tumors using CNN. According to the need for early detection of melanoma and the increasing cost of ways to diagnose the disease, the present study tries to provide a more accurate and cost-effective method based on AI for recognizing malignant skin lesions. The scholars utilized the CNN technique on the basis of deep learning technique to identify, classify, and segment skin lesions that are malignant. The results obtained from the performance of the presented technique displayed that the CNN procedure on the basis of the deep learning procedure with 89.5 % accuracy was able to diagnose skin disease, which is a significant amount.

Banerjee et al. [21] diagnosed malignant skin tumors using deep learning and fuzzy logic techniques. Abnormal division of skin cells causes melanoma due to exposure of the skin to UV rays. Due to the dangerousness of this type of cancer, timely identification of the illness has the potential to reduce the time of the cure process. Deep CNNs have been applied in this paper to detect malignant skin blemishes. This technique is an advanced computational method for classifying, identifying, and classifying skin spots in disease detection. The computational method was tested on 20,250 images of skin blemishes. The results obtained from the efficiency of the computational approach illustrated this approach possesses 79.84 % accuracy in the Jac data set, 86.99 % accuracy in the ISIC 2019 data set, and 88.6 % accuracy in the PH^2^ set of data. The values achieved by the data set indicated that the suggested computational approach gives a good capability in diagnosing the disease.

### 1.3 Motivations and contributions

Based on the literature, various kinds of methods were performed in this respect. Nevertheless, metaheuristic-based strategies provide finer outcomes compared to the other techniques. The current research suggests a novel method to detect melanoma cancer by the use of learning through reinforcement, extraction of feature, selection of feature, and SVM. The method uses reinforcement learning for segmenting the skin regions, followed by the extraction and selection of useful features using the Enhanced Fish Migration Optimizer (EFMO) algorithm. Then, the outcomes are categorized on the basis of an optimized SVM based on the EFMO algorithm. The key implications of the current essay have been found to be.

• The use of reinforcement learning for skin region segmentation, which is a novel approach in melanoma detection.
• The application of the EFMO algorithm for feature extraction and selection has not been used in previous studies on melanoma detection.
• The optimization of support vector machines using the EFMO algorithm, which leads to finer efficiency in comparison with traditional approaches.
• The validation of the proposed method using the Melanoma dataset of SIIM-ISIC and a juxtaposition with 12 further methods, show that the proposed method outperforms the others.

RETRACTED

## 2 Materials and methods

Dermoscopic images are widely used in diagnostic fields, and the application of intelligent methods can significantly improve the speed and accuracy of data analysis. In this section, we introduce preprocessing, which involves dividing the image into sub-images. Previous research in medical image segmentation has not given much attention to the impact of sub-image dimensions on the resulting image segmentation. To address this gap, we propose a multifactorial structure to select the most appropriate dimensions for the sub-images. In this paper, a thorough explanation of the methodology and operation of this method are provided.

Next, the reinforcement learning approach is applied to perform image segmentation. This section introduces the modes, actions, and rewards used in the reinforcement learning algorithm. Following this, the post-processing step enhances the excellence of the segmented picture using morphological operators. The most appropriate dimensions for these operators are determined through the use of the trial-and-error method. Finally, the paper presents the practical outcomes of picture segmentation utilizing the reinforcement learning approach for distinct mode categories.

The method of learning through reinforcement for segmentation of picture in dermoscopy involves two primary stages: training and testing. while the stage of the training, the model uses physically images segmented to acquire the appropriate variables for image segmentation utilizing the reinforcement learning method. At the end of the training stage, a strategy table is generated that contains the optimal values of actions for each case. In addition, the most suitable dimensions of the images and the size of the morphological operators for enhancing the excellence of the image segmented are determined in this section.

RETRACTED

In the testing stage, the information obtained from the training stage is used to segment new images. Fig. (1) provides a block diagram of the processes involved in the training phase.

**Fig. 1:** Block diagram of the processes in the training phase.

Overall, the proposed method involves a supervised learning approach, where the system learns from the manually segmented images to develop an optimal strategy for image segmentation. This approach can significantly enhance the efficacy and accuracy of dermoscopic image analysis; moreover, the results of this study demonstrate its effectiveness in accurately segmenting dermoscopic images.

### 2.1 Pre-processing process

The process includes two parts, which are filtering and dividing the image into a set of sub-images. Filtering gives a smoother image than the original image by reducing the effect of noise. Eq. (1) shows the mathematical expression filtering.

(1) $$\forall p_{ij}\in I,N_{n}=\left[p_{ij}^{*}|\;dist\left(p_{ij},p_{ij}^{*}\right)<n\right]$$

here, I defines the matrix of the amounts of the image intensity and $p_{ij}$ is the pixel in the $i^{th}$ row and $j^{th}$ column of the intensity matrix. A neighbor of pixel p can be defined by $N_{n}$, where, $P^{*}$ describes the pixel neighboring to p in the distance n.

To send images for more processing, the basic image is split into a group of $\left(L_{i},w_{i}|i=1,2,\ldots ,m\right)$ images. To determine the most appropriate dimensions of the images, a multifactorial structure is performed according to Fig. (2).

**Fig. 2:** Multi-factor structure arrangement.

This structure consists of a set of reinforcement learning factors with the agent symbol $Agent_{i}$, i=1,2,…,m and a controlling factor with the symbol $Agent_{c}$. Each reinforcing learning factor in the image-processing process segments the $k^{th}$ sub-picture; moreover, it leads the coefficient of dissimilarity $D_{i}\left(k\right)$ to the control agent. If $Agent_{j}$ increases in the segmentation of the three consecutive images, or if $Agent_{j}$ is large at the end of the distortion, the coefficient of inequality $D_{ij}\left(k\right)$ is eliminated by the control agent. The relation related to the performance of the control agent is shown in Eq. (2). The deleted factor is indicated by the expression *killed* in this relation.

(2) $$Agent_{j}\to killed\Rightarrow \left\{ \begin{array}{c} D_{ij}\left(k\right)>D_{ij}\left(k-1\right)>D_{ij}\left(k-2\right)\\ D_{ij}\left(k\right)=\max_{z=1,2,\ldots ,m}\left(D_{iz}\left(k\right)\right) \end{array}\right.$$

Eq. (3) represents the mathematical expression for the values of the dissimilarity coefficient $D_{i}$.

(3) $$D_{i}=\frac{\sum_{i=1}^{M}\sum_{j=1}^{N}XOR\;\left(I,I_{d}\right)}{r_{I}\times c_{I}}$$

where, I is the binary value of the image resulting from the segmentation by the reinforcement learning factor, I, represents the binary values resulting from the segmentation of the image manually, and the values M, N, $r_{I}$ and $c_{I}$, represent the pixels' number in the rows and columns and the rows' number and columns in the image, respectively.

RETRACTED

However, the modern trend in the different imaging fields can be considered also in this sense to guarantee remarkable classification performances [22,23].

### 2.2 Processing process

In the current process, the picture has been segmented utilizing the thresholding operator, then the resulting image is processed using the open morphology operator [24]. The reinforcing learning factor obtains the threshold and radius values of the morphology operator for each sub-image (which includes different fragments of the processed divided image) using the Learning-Q learning algorithm. The processed image's block diagram is shown in Fig. (3).

**Fig. 3:** Block diagram of the processed image.

In this process, the values of the actions, which are denoted by the set δ, and its members are arranged in pairs of intensity values $\tau_{i}$, which are selected from the minimum value of intensity in the image below with $g_{\min}$ representation and the maximum value of intensity in the image below with the representation $g_{\max}$, and the values of the radius. The operator $\nu_{j}$ has been chosen through the intended values of $v_{l}$ as well as $v_{m}$. Eq. (4) displays the set δ.

(4) $$\delta =\left[\left(\tau_{1},\nu_{1}\right),\left(\tau_{1},\nu_{2}\right),\ldots ,\left(\tau_{i},\nu_{j}\right)\right]$$

The vector S is used to display the states according to Eq. (5). The components of this vector include area, compactness, the quantity of objects in the segmented image, and the spatial position of the picture, which have been represented by $X_{1}$, $X_{2}$, $X_{3}$, $X_{4}$, respectively. In Eq. (5), the state vector is denoted by the symbol S:

(5) $$S=\left[X_{1},X_{2},X_{3},X_{4}\right]$$

The reward values are denoted by R. To obtain the reward values according to Eq. (6), the dissimilarity coefficients are compared in two consecutive repetitions, and based on the result of this comparison, one of the values r and j are attributed as a reward to the reinforcement learning factor.

(6) $$R=\left\{ \begin{array}{c} R_{1},D_{I}^{after}<D_{I}^{before}\\ R_{2},otherwise \end{array}\right.$$

The major target of the post-processing process is enhancing the fragmented picture's quality in the processing stage by using the morphology operators to open and close and determine the most appropriate dimensions for these operators.

RETRACTED

Trial and error methods are used to determine the most appropriate dimensions for morphological operators. After splitting the base image of different values of $\lambda_{i}=1,2,\ldots ,m$, which are considered as the radius i of the disk-shaped morphology operators, $\lambda^{*}$ corresponds to the lowest dissimilarity coefficient of $D_{i}$ is considered as the radius of these operators in the test stage. $\lambda^{*}$ has been obtained via the subsequent formula:

(7) $$\lambda^{*}=\arg\min_{i}D_{i}$$

Table 1indicates the values of the two categories of states for which the program has been executed (see Table 2).

**Table 1:** Values of the two categories of states for which the program.

States	Mode 1	Mode 2
	Number of states	Number of states
$X_{1}$	9	4
$X_{2}$	5	4
$X_{3}$	4	3
$X_{4}$	4	3

**Table 2:** Parameter values of the algorithms throughout the comparison.

Algorithm	Parameter	Value
Billiard-based Optimization algorithm [25]	Number of pockets	22
	w	0.7
	ES	0.3
WHO [26]	$\alpha_{1}$	0.9
	$\beta_{1}$	0.3
	$\alpha_{2}$	0.2
	$\beta_{2}$	0.8
LOA [27]	Number of Prides	5
	Percentage of Nomad Lions	0.3
	Roaming Percentage	0.4
	Probability of Mutate	0.1
	Mating probability	0.4
	Rate of Sex	0.85
	Rate of Immigrate	0.5
FMO [28]	α	0.15

**Table 3:** The structure of the applied system.

Name	Setting
Programming software	MATLAB R2019b
Hardware	Intel® Core™ i7-4720HQ
System of Operation	Windows 10
RAM	16 GB
CPU	1.60 GHz
Frequency	1.99 GHz

In the form of the images obtained from image segmentation by the reinforcement learning method, the best results for Mode 1 and Mode 2 have been illustrated by Fig. 4(A–C).

**Fig. 4:** Some examples of the process for (A) original image, (B) Mode 1, (C) Mode 2.

### 2.3 Features extraction

This process aims to create raw data applicable for later statistical processes, which is a usual procedure in various kinds of data processing like audio processing, image processing, etc. This is related to choosing a feature to explain the image with less information. The included properties of features must be described with a group of unique features [29]. For example, in the image of people's faces, the distance between the eyebrows is a suitable feature that must be extracted. In this study, we utilize feature extraction to benefit from its advantages and for providing more accurate outcomes. The current research uses feature extraction for obtaining valuable data from the input images [30]. For this purpose, several features have been utilized. In the current investigation, some different characteristics were used from statistical features, texture features, as well as geometric characteristics. These features' formulation is given in the equations [[8], [9], [10], [11], [12], [13], [14], [15], [16], [17], [18], [19], [20], [21], [22], [23], [24]]:

(8) $$Rectangularity=\frac{Area}{a\times b}$$

(9) $$Elongation=\frac{2\sqrt{Area}}{a\sqrt{\pi }}$$

(10) $$Area=\sum_{i=1}^{M}\sum_{j=1}^{N}p\left(i,j\right)$$

(11) $$Form\;factor=\frac{Area}{a^{2}}$$

(12) $$Solidity=\frac{Area}{ConvexArea}$$

(13) $$Irregularity\;index=\frac{4\times \pi \times Area}{Perimeter^{2}}$$

(14) $$Perimeter=\sum_{i=1}^{M}\sum_{j=1}^{N}b_{p}\left(i,j\right)$$

(15) $$Eccentricity=\frac{2}{a}\times \sqrt{\left(a^{2}-b^{2}\right)}$$

(16) $$\text{Contrast}=\sum_{i=1}^{M}\sum_{j=1}^{N}p^{2}\left(i,j\right)$$

(17) $$\text{Energy}=\sum_{i=1}^{M}\sum_{j=1}^{N}p^{2}\left(i,j\right)$$

(18) $$\text{Homogeneity}=\sum_{i=1}^{M}\sum_{j=1}^{N}\frac{p\left(i,j\right)}{1+\left|i-j\right|}$$

(19) $$\text{Correlation}=\sum_{i=1}^{M}\sum_{j=1}^{N}\frac{p\left(i,j\right)-\mu_{r}\mu_{c}}{\sigma_{r}\sigma_{c}}$$

(20) $$\text{Mean}=\frac{1}{MN}\sum_{i=1}^{M}\sum_{j=1}^{N}p\left(i,j\right)$$

(21) $$\text{Entropy}=-\sum_{i=1}^{M}\sum_{j=1}^{N}p\left(i,j\right)\log\;p\left(i,j\right)$$

(22) $$\text{Variance}=\frac{1}{MN}\sum_{i=1}^{M}\sum_{j=1}^{N}\left(p\left(i,j\right)-\mu \right)$$

(23) $$Std=Variance^{2}$$

Invariant moments:

(24) $$\varphi_{1}=\eta_{20}+\eta_{02}\;\varphi_{2}={\left(\eta_{20}-\eta_{02}\right)}^{2}+4\eta_{11}^{2}\varphi_{3}={\left(\eta_{30}-3\eta_{12}\right)}^{2}+{\left(3\eta_{21}-\mu_{03}\right)}^{2}$$

In the above equations:

a: Major axis

b: Minor axis

$b_{p}$: Exterior side size of the border pixel

p(i,j): The value of pixels intensity at (i,j).

RETRACTED

*MN*: The image size.

μ: Mean value of pixels

σ: StD of pixels

However, feature extraction extracts significant information from the image, some of them may have useless or so low information for a definite case that can be neglected. In this study, to eliminate such features, a metaheuristic-based methodology has been proposed. To find the best features among all, a cost function should be utilized. The main objective is minimizing the integration function based on the multiplication, including accuracy of categorization and F-score. The cost function is given below:

(25) $$\mathrm{Cos}\;t_{j}=\alpha \times accuracy_{j}+\beta \times \frac{\sum_{j=1}^{M_{b}}F\left(FS\left(j\right)\right)}{\sum_{j=1}^{N_{b}}F\left(k\right)}$$

where, $accuracy_{i}$ describes the classification accuracy rate and is achieved as equations [30,28]:

(26) $$accuracy_{j}\left(N\right)=\frac{\sum_{j=1}^{\left|M\right|}assess\;\left(m_{i}\right)}{\left|M\right|},m_{i}\in M$$

(27) $$assess\left(m\right)=\left\{ \begin{array}{c} 1,if\;classify\;\left(m\right)=mc\\ 0,otherwise \end{array}\right.$$

where, M defines the number of test sets, mc shows the class of item m.

on the other hand, F1-score measures the discrimination of two sets of actual-valued. By taking into consideration the vectors of training $X_{k},k=1,2,\ldots ,m$. Assuming the quantity of positive ($n^{+}$) and negatives ($n^{-}$) sample, the $i^{th}$ feature's F-score has been illustrated in equation (28) way:

(28) $$F\left(j\right)=\frac{{\left({\bar{x}}_{j}^{+}-{\bar{x}}_{j}\right)}^{2}+{\left({\bar{x}}_{j}^{-}-{\bar{x}}_{j}\right)}^{2}}{\frac{1}{m^{+}-1}\sum_{k=1}^{n^{+}}{\left({\bar{x}}_{k,j}^{+}-{\bar{x}}_{j}^{+}\right)}^{2}+\frac{1}{m-1}\sum_{k=1}^{n^{-}}{\left({\bar{x}}_{k,j}^{-}-{\bar{x}}_{j}^{-}\right)}^{2}}$$

where, α+β=1. Here, α=0.65 and β=0.35, F(FS(i)) determines the application for evaluating the current score of characteristics, and, ${\bar{x}}_{j}$, ${\bar{x}}_{j}^{-}$, ${\bar{x}}_{j}^{+}$ represent, in turn, $i^{th}$ feature's mean value of the set, datasets of positive, and negative, ${\bar{x}}_{k,j}^{-}$ and ${\bar{x}}_{k,j}^{+}$ define the $j^{th}$ attribute of the $k^{th}$ positive and negative samples. So, the $j^{th}$ feature's F-score has been achieved in equation (29) way:

(29) $$F_{i}=\frac{\sum_{i=1}^{l}{\left({\bar{x}}_{j}^{i}-{\bar{x}}_{j}\right)}^{2}}{\sum_{i=1}^{l}\frac{1}{m_{i}-1}\sum_{k=1}^{n_{i}}{\left({\bar{x}}_{k,i}^{i}-{\bar{x}}_{i}^{j}\right)}^{2}}$$

Where, ${\bar{x}}_{j}$, ${\bar{x}}_{j}^{i}$ illustrate the feature number's mean value, j for the entire dataset and i for the dataset quantity, and ${\bar{x}}_{k,i}^{i}$ defines the attribute number j of the instance number j.

The subsequent proportion is evaluating the scores of the feature masks. FS(i) is achieved as equation (30):

(30) $$FS\left(i\right)=\left\{ \begin{array}{c} instance\;j,if\;j\;is\;selected\\ 0,if\;j\;is\;not\;selected \end{array}\right.$$

The main idea for feature classification in this study is to minimize Eq. (25)

### 2.4 Enhanced fish migration optimization algorithm

#### 2.4.1 Introduction

Although fish pursue various goals by swimming in the water, fish migration optimization is inspired by the migrating grayling mechanism. The cycle of life has been shown in the following figure and the various age levels within five years are indicated by '0+' to '4+', fertility of individuals returning to their birthplace is represented by 'P2′ to 'P4′, and 'S1′ to 'S4′ determines the number of individuals who survived. '0+' specifies the nascent fishes and they do not migrate to find food and do not move away from their place of birth and look for food around the place of birth. Over time, as graylings grow, they can migrate and find more distant food, but when they reach the stage of '4+', they must return to where they were born. Also, natural enemies eat several graylings every year. Fig. (5) illustrates the cycle of fish Life.

RETRACTED

**Fig. 5:** Cycle of fish Life.

#### 2.4.2 Initializing

For optimization, the fish's location occurs randomly within five steps of age. The proportion of graylings' numerals have been indicated by seq and this ratio is 1: 1: 1: 0.66: 0.66. the capability of immigration is expressed by z_eng. The primary value of individual grayling is 2.

#### 2.4.3 Evolution

From the '2+' stage, the graylings commence migrating. The fish's power for migrating has been achieved from equation (31) formula based on their energy.

(31) $$Z_{eng\left(j\right)}=Z_{eng\left(j\right)}-\frac{f_{j}}{\sum_{j=1}^{n}f_{j}}$$

Where j indicates the j−th fish, the number of fishes is specified by n, of the cost function's value for jth fish has been illustrated by $f_{j}$.

Discovering a finer solution can expand the fish's power, but as the fish ages, the fish's energy reduces. [Equation (32)].

(32) $$Z_{eng\left(j\right)}=Z_{eng\left(j\right)}+r1*Z\_eng\left(j,init\right)$$

Where r1 defines an amount randomly in the range [0,1], and the initial energy of j is indicated by $Z_{eng}\left(j,init\right)$.

#### 2.4.4 Fecundity

Given that fish may be eaten by enemies, their number decreases over time, the corresponding equation (33) is presented below:

(33) $$Z_{number\left(t+1\right)}=Z_{number\left(t\right)}*state\left(t\right)$$

The number of grayling at the (t+1)−th phase is represented by Z_number(t+1). The survival proportion is expressed by stat which is 1: 0.93: 0.91: 0.37: 0.66 from the first stage to four. All fishes survive at the '0+' step but many of them die in the '4+' stage. The goal is to increase the ability to explore and prevent the algorithm from localizing. To keep the number of the fish constant, newborn fish substitutes dead fish, and the surviving fish reposition is founded on the optimal solution (equations [31,32]).

(34) $$temp=r2*\left(Z_{v}-gb_{pos}\right)$$

(35) $$Z_{v}=temp+gb_{loc}$$

Where r2 indicates an amount randomly in the range [0,1] and the surviving fish is specified by $Z_{v}$, $gb_{loc}$ represents the location of the global optimum.

#### 2.4.5 Motion

Fish move or migrate in old age (equations [[33], [34], [35]]).

(36) $$ori_{speed}=\left\{ \begin{array}{c} Z\left(j\right)-Z\_pre\left(j\right)\;if\left(r3\geq 0.5\right)\\ Z\_pre\left(j\right)-Z\left(j\right)\;else \end{array}\right.$$

(37) $$Z\left(j\right)=ori_{speed}*consumption+Z_{eng\left(j,init\right)}*r4*\left(gb_{pos}-Z\left(j\right)\right)$$

(38) $$consumption=\left\{ \begin{array}{c} Z_{eng}\left(i,init\right)*r4\;if(Z\_eng\left(j\right)\geq Z_{eng}\left(j,\mathrm{int}\right)\\ Z_{eng}\left(j\right)*r6\;else \end{array}\right.$$

where, r3,r4,r5, and r6 are amounts randomly in the range [0,1]. The earlier location of j is specified by $Z_{pre}$, consumption is the kinetic energy of motion, and it is defined by $Z_{eng}$. The location update in stages '0′, '1′ as well as '4′ is obtained through equation (35) and the location update in stages '3′ and '2′ is obtained through equation (37).

RETRACTED

#### 2.4.6 Enhanced Fish Migration Optimizer

The Fish Migration Optimizer (FMO) is a new metaheuristic optimizer that by considering a novel metaheuristic, has excruciatingly great outcomes for various kinds of objective functions based on [28]. The reference shows that this algorithm provides well-organized results for optimization [14,[36], [37], [38], [39]]. However, in some cases, the original FMO Algorithm may have been trapped in the local optimal point and delivered unpromising results with lower convergence speed [40]. Here, an improved model of the Fish Migration Optimization is made and utilized for optimal feature classification purposes.

One enhancement is to utilize an approach, which is on the basis of the OBL (Opposition-based Learning). The Opposition-based Learning method with higher investigation of the solution space, delivers promising achievements to modify the productivity of the optimization algorithms [41]. This technique first forms the complement value of each of the randomly generated candidates and then, by comparing each of the candidates with their complement value, the optimum candidate is chosen as the new one and the other one has been removed. To make a compliment candidate, $Z_{eng\left(j\right)}^{new}$, the complement value is obtained as below:

(39) $$Z_{eng\left(j\right)}^{new}=Z_{eng\left(j\right)}^{\max}+Z_{eng\left(j\right)}^{\min}-Z_{eng\left(j\right)}$$

where, $Z_{eng\left(j\right)}^{new}$ refers to the opposed location of $Z_{eng\left(j\right)}$, and $Z_{eng\left(j\right)}^{\min}$ and $Z_{eng\left(j\right)}^{\max}$ depict the solution's upper and lower boundaries, respectively. Here, 30 % of the primary population has been obtained by the aforementioned method.

The subsequent mechanism is to utilize the theory of Chaos to provide a better result in terms of convergence speed. The chaos theory employs a chaotic plan to produce pseudo-stochastic individuals in place of stochastic individuals [[31], [32], [33], [34]]. This mechanism employs several maps to reduce the complexity of the algorithm and likewise to escape from the local optima. The present investigation employs the Sine plan for enhancement. The aforementioned map is a unimodal map that can be formulated as equation (40):

(40) $$r_{i+1}=\frac{\gamma }{4}\times \sin\left(\pi r_{i}\right),r\in \left[0,1\right]\;0<\gamma \leq 6$$

Here, γ=4 [35]. The histogram value of the mechanism has been shown in Fig. (6).

RETRACTED

**Fig. 6:** PDF of the Sine map.

#### 2.4.7 Confirmation

To authenticate the efficiency of the suggested Enhanced Fish Migration Optimizer, it has performed some standard performance indices and the accomplishments are validated accompanying some newest techniques, comprising BOA (Billiard-based Optimization Algorithm) [25], WHO (Wildebeest Herd Optimization) [26], Lion optimization algorithm (LOA) [27], as well as the original Fish Migration Optimizer (FMO) [28] to determine its to show its accuracy and precision and to show its efficiency in a reasonable position. The following table shows the parameter values of the optimization algorithms by comparing them.

All of the simulations were performed by MATLAB 2018b. The maximum iteration value and the optimizer's population size have been found to be, in turn, 200 and 70, and all of the optimizers for each benchmark function are performed 30 times independently. The mentioned settings are performed to provide fair validation. The structure of the applied model has been illustrated in the following table.

The equation of mathematics of the studied test functions has been defined in the following way.

The first function is Rotated High Conditioned Elliptic. The minimum value of this function is 100 and its mathematical formula is as equations [[27], [42], [43], [44]]:

(41) $$F_{1}\left(x\right)=f_{1}\left(M\left(x-o_{1}\right)\right)+F_{1}^{*}$$

The next function utilized in this study is the Rotated Bent Cigar. This function possesses a 200 minimum value; moreover, it can be obtained as below:

(42) $$F_{2}\left(x\right)=f_{2}\left(M\left(x-o_{2}\right)\right)+F_{2}^{*}$$

Here, the lowest value of the mentioned exam function has been found to be 200.

Another equation is Rotated Discuss which possesses a 300 minimum value. The equation of this application has been given below:

(43) $$F_{3}\left(x\right)=f_{3}\left(M\left(x-o_{3}\right)\right)+F_{3}^{*}$$

The final benchmark function in this assessment is Rotated and shifted brock. The minimum value of this study is 400 and is calculated as below:

(44) $$F_{4}\left(x\right)=f_{4}\left(M\left(\frac{2.048\left(x-o_{4}\right)}{100}\right)+1\right)+F_{4}^{*}$$

Four measurement indicators, the Minimum, Maximum, STD (Standard Deviation), and Mean values are used to analyze the analyzed metaheuristics. The outcomes of the juxtaposition of the proposed Enhanced Fish Migration Optimization algorithm with the analyzed metaheuristics have been recorded in the following table.

RETRACTED

As can be derived through the findings of the table above, the proposed EFMO optimization algorithm gives the optimum results for the four studied test functions for all minimum values, average amount, and max amount after 30 times autonomous administrations. This indicates that the proposed approach conveys the optimum efficiency as concerns precision. Also, based on the standard deviation of the outcomes during 30 time administrations, it has resulted that the suggested technique provides a more reliable solution for the problem than all of the additional proportional approaches. The outcomes also illustrate there is a trade-off between time and accuracy when using the proposed EFMO algorithm. While the system's running time is slower than the original version due to the added improvements, the increase in accuracy outweighs the slight decrease in speed. This trade-off is negligible since the difference in running time is relatively small.

#### 2.4.8 Time complexity

The proposed method's time complexity for performing clustering is expressed as follows.

1. The quantity of performances to initialize distinct variables has been found to be 1 time; therefore, the period complication of stage (1) has been found to be O(1).
2. The Enhanced Population of Fish must conduct *N* operations to initialize the primary location randomly. So, the time complication of stage (2) has been found to be O(N+N).
3. Upgrade the location of the mayflies, and the quantity of performances also needs *N* times. so, the time complication of stage (3) has been found to be O(N+N).
4. The quantity of performances organized in accordance with the present value of Fish fitness is *2Nlg2N*, so the complication of time of stage (4) has been found to be O(2Nlg2N).

After the above steps, the complication of time of the DESMA optimizer after NC iterations is O(2N+2+2Nlg2N).

#### 2.4.9 EFMO algorithm for feature selection

Based on the result, we have decided to use this algorithm for minimizing Eq. (25). The optimization algorithm has the potential to be defined in the subsequent pseudo-code.

(1) Commence
(2) Initialization of the EFMO variables for the problem based on section (2.4)
(3) Performing EFMO to Eq. (25) as well as evaluating value of cost
(4) Updating the EFMO to achieve the finest lowest value
(5) Examining criteria of stopping: if stopping criteria are not met, examine (3), otherwise, examine (5)
(6) Illustrating the chosen optimal attributes
(7) End

RETRACTED

### 2.5 Categorization of the features on the basis of the SVM (support vector machines) optimized by EFMO

Support Vector Machines has been counted as a controlled learning optimizer to be utilized for regression and classification problems; nevertheless, commonly has been utilized in classification issues. In this optimizer, on the data scatter diagram, each data sample has been strategized as a point in the nD space (n defines the properties number that a data sample has) and the amount of each data attribute is one of the coordinate points on the curve. Thus, through straight line drawing, it classifies various and separate data. Simply put, support vectors are the coordinates of a single observation. An SVM is a boundary that optimally split data collections. Support Vector Machine specifies the best decision surface to data as follows:

(45) $$y=sgn\left(\sum_{i=1}^{M}y_{i}\alpha_{i}K\left(z,z_{i}\right)+b\right)$$

Where, z describes a set vector of d−Dd test, $z_{i}$ expresses the number of set vector of training i, M refers to the numbers of the training set, y signifies a class label between −1 and 1, b and $\alpha =\left[\alpha_{1}\ldots \alpha_{N}\right]$ have been defined as the system variables, and K describes the kernel application.

Here, Support Vector Machine is utilized to classify melanoma in two categories of non-cancerous and cancerous classes. Different kernel functions are introduced for the optimal designing of the SVM. An extensively utilized functions kernel is the RBKF (Radial Basis Kernel function). This has been mostly used due to its ability for multi-dimensional data classification. However, this kernel has fewer setting parameters than a polynomial kernel, it has similar in efficiency to the other kernels. Therefore, it is an efficient option that is used here for the designed SVM.

There are two parameters in the RBF-based support vector machine (C and γ) that have a good effect on its efficacy. The variable C is an adjusting variable for the support vector machine, where, changes the categorization samples of training by increasing the function margin of decision to the maximum amount. Generally, the tiny dimensions of C improves the straightforward function of decision. Also, the parameter γ as the other parameter defines the effect of distance for a sample of single training. A smaller value of this parameter defines the far effect of the exercise example, and it comes true for the opposite one as well.

It illustrates optimal selection of the γ and C is too essential for efficient designing of the SVM. Different studies have been done for this purpose to provide the best optimal values of these parameters [42]. The best condition happens when the performance of parameter selection has been maximized. In the current investigation, the designed EFMO has been employed for the optimal selection of C and γ. The method of optimizing the SVM based on the two parameters is a two-folded approach.

RETRACTED

At first, the γ value has been adapted based on the optimal accuracy value by defining a route by the EFMO algorithm. After randomly initializing and achieving the optimal value of the parameter γ and assuming parameter C, the best value for the parameter γ has been achieved. Afterward, the optimal value of parameter γ is considered as constant and the EFMO algorithm is evaluated for achieving the best C value. then, the best value of these two parameters is achieved for classification. The workflow of the suggested optimized SVM is depicted in Fig. (7).

**Fig. 7:** The workflow of the suggested optimized SVM.

## 3 Discussions and simulations

In the current phase, the efficacy of the utilized methodology for melanoma diagnosis have been discussed. To provide this validation, we need a study case. In this study, we employed the SIIM-ISIC melanoma dataset for method authentication. The technique is then hold compared to some the most novel strategies that have been found to be CNN [43], Side-by-Side technique [44], Fractal analysis [45], GA [46], SVM [47], Fusion method [48], Delaunay Triangulation [49], texture Descriptor of MED-NODE [50], color descriptor of MED-NODE [50], Spotmole [51], ResNet-101 [52] for more clarification.

### 3.1 Dataset

In this study, we use a skin cancer collection, called SIIM-ISIC Melanoma dataset for validation of the suggested melanoma diagnosis system. This SIIM-ISIC Melanoma dataset is a well-known dataset for medical imaging. All of the images were produced in DICOM layout that should be extracted by famous archives and comprise metadata and image. The collection includes JPEG and TFRecord formats. The input images are of size 1024 × 1024. Fig (8) shows some examples of this dataset.

**Fig. 8:** Several instances of the Melanoma dataset of SIIM-ISIC.

The aforementioned dataset might be downloaded via the following hyperlink: https://www.kaggle.com/c/siim-isic-melanoma-classification.

### 3.2 Model evaluation

The suggested method contains three main steps for diagnosis. At first, we used reinforcement learning to segment the texture of the skin in the input images. Afterward, a new metaheuristic method has been applied for classification and extracting features. The proposed algorithm is named Enhanced Fish Migration Optimization algorithm which shows good results based on validations. This algorithm is then utilized for feature selection of the extracted features from the segmented images. Finally, the algorithm is used for the optimal designing of an SVM for classifying the cancerous pictures. The model has been validated on the basis of several metric indexes, which are Specificity (%), Accuracy (%), PPV (%), NPV, and Sensitivity. In summary, sensitivity, accuracy, NPV, PPV, and specificity are important classification indexes utilized to assess the efficiency of a categorization system. Mathematically, the model formulation of these indexes can be defined as follows:

(46) $$Sensitivity=\frac{correctly\;detected\;skin\;cancer\;cases}{Total\;skin\;cancer\;cases}$$

(47) $$Specificity=\frac{correctly\;detected\;healthy\;skin\;cases}{total\;healthy\;skin\;cases}$$

(48) $$accuracy=\frac{correctly\;detected\;cases}{total\;cases}$$

(49) $$PPV=\frac{correctly\;detected\;skin\;cancer\;cases}{detected\;skin\;cancer\;cases}$$

(50) $$NPV=\frac{correctly\;detected\;healthy\;skin\;cases}{detected\;healthy\;skin\;cases}$$

Sensitivity, accuracy, Positive Predictive Value (PPV), Negative Predictive Value (NPV), and specificity are performance metrics utilized in categorization troubles. Accuracy assesses the ratio of properly categorized samples out of the entire ones, sensitivity assesses the ratio of TP instances out of the total positive instances, specificity measures the proportion of true negative samples out of the entire negative ones, and PPV assesses the ratio of TP instances out of the total predicted positive instances, while NPV evaluates the ratio of TN samples out of the total predicted negative samples (see Table 4).

RETRACTED

As mentioned before, the proposed method is compared with 10 other methodologies to provide better validation. Table 5 indicates the performance evaluation of the recommended strategy and the other compared techniques.

**Table 4:** The outcomes of the juxtaposition of the proposed Enhanced Fish Migration Optimization algorithm with the analyzed metaheuristics.

Test Function	Index	BOA [25]	WHO [26]	LOA [27]	FMO [28]	EFMO
($F_{1})$	Max	3.251E+05	8.234E+05	4.267E+04	6.821E+03	1.013E+03
	Min	2.264E+05	5.394E+05	3.134E+04	5.218E+03	2.162E+03
	Mean	3.238E+05	6.814E+05	4.356E+04	5.113E+04	2.142E+04
	STD	4.236E+05	5.217E+05	3.923E+04	4.156E+04	2.211E+04
	Time (s)	14.11	13.15	13.08	12.82	13.49
$\left(F_{2}\right)$	Max	5.354E+04	2.935E+04	1.137E+04	6.128E+03	3.138E+03
	Min	3.208E+04	3.551E+04	2.689E+04	2.374E+03	2.145E+03
	Mean	4.256E+04	3.743E+04	1.468E+04	4.636E+03	2.137E+03
	STD	4.121E+04	3.381E+04	2.089E+04	2.439E+03	2.024E+03
	Time (s)	12.92	12.67	10.95	10.17	11.81
$\left(F_{3}\right)$	Max	7.328E+03	6.357E+03	8.294E+02	9.291E+01	5.183E+01
	Min	5.641E+03	4.284E+03	7.228E+02	6.934E+01	3.954E+01
	Mean	6.394E+03	5.671E+03	7.266E+02	7.653E+01	4.563E+01
	STD	6.181E+03	5.492E+03	7.129E+02	7.537E+01	4.461E+01
	Time (s)	10.90	9.67	8.50	7.66	8.01
$\left(F_{4}\right)$	Max	8.394E+03	6.927E+02	4.534E+02	3.294E+01	2.643E+01
	Min	5.186E+03	3.039E+02	3.394E+02	2.168E+01	1.735E+01
	Mean	5.285E+03	6.528E+02	6.364E+02	5.176E+01	2.434E+01
	STD	4.637E+02	5.236E+02	3.135E+02	4.549E+01	5.674E+01
	Time (s)	14.22	13.83	11.74	9.28	11.57

**Table 5:** Performance evaluation of the recommended strategy and the other compared techniques.

Technique	Metric of Performance				
	Accuracy	Sensitivity	Specificity	PPV	NPV
Fractal analysis [45]	81.66	90.83	81.66	73.33	85.83
CNN [43]	78.33	75.83	56.66	61.66	76.66
Delaunay Triangulation [49]	80.00	82.50	80.00	72.50	82.50
Side-by-Side method [44]	60.83	78.33	51.66	51.66	73.33
Genetic Algorithm [46]	73.33	73.33	73.33	72.50	78.33
Fusion method [53]	83.33	73.33	70.83	63.33	73.33
SVM [54]	78.66	78.33	70.83	68.33	73.33
MED-NODE texture Descriptor [50]	66.66	81.66	73.33	75.83	73.33
MED-NODE color descriptor [50]	70.83	68.33	60.83	79.16	70.00
Spotmole [50]	75.83	56.66	56.66	80.83	64.16
ResNet-101 [55]	80.00	72.50	72.50	85.00	80.83
Proposed Method	85.00	85.00	86.66	81.66	87.50

According to Table 5 that the proposed strategy with 85 % accuracy suggests the highest efficacy than the juxtapositional methodologies. Likewise, with an 85 % sensitivity value for the suggested methodology which is uppermost toward the newest techniques it indicates the reliability of the suggested technique. This is also proved by PPV, specificity, and NPV values. The finer amount of PPV and NPV for the proposed technique delivers well probability results of it in diagnosing cancer against the other techniques. Finally, well achievements of the specificity for the suggested technique along with its sensitivity indicate its higher prevalence-independent results. We also analyzed the Region of Convergence (ROC) curve based on values of metric achieved to assess the efficiency of the study. The Region of Convergence is an extensively-utilized measurement technique to assess the efficiency of any categorization system. The area below the ROC graph defines the effectiveness of the methods, where, by closing the AUC to 1, it shows its higher classification ratio. Fig. (9) shows the ROC curve of the approach toward the others.

**Fig. 9:** The ROC curve of the method toward the others.

It can be witnessed through the outcomes of Fig. (9), the ROC value of the recommended technique is so proper toward the other techniques that shows its higher efficiency for classification toward the others. Accordingly, the suggested technique delivers significantly effective achievements for melanoma diagnosis.

RETRACTED

While the proposed method for the optimum detection of melanoma cancer is a valuable contribution to the field, some limitations should be acknowledged. Firstly, the study uses a specific dataset, for validating the proposed method, which is normal. While the dataset is widely used in the research community, it may not be representative of the full range of melanoma cases that exist in the real world. Future research could focus on testing the suggested approach on datasets, which are more distinct and larger to further certify its efficiency and generalizability. Secondly, the proposed method only utilizes visible light images for melanoma diagnosis and does not incorporate other imaging modalities such as infrared or ultrasound imaging. While the method achieves good results with visible light images, integrating information from multiple imaging modalities could enhance the reliability and accuracy of the diagnosis. Thirdly, the suggested method only focuses on the segmentation and classification of melanoma lesions and does not take into account other clinical factors such as patient history, demographics, or other clinical data. Incorporating additional clinical data could further improve the accuracy of the diagnosis and enable more personalized and effective treatments. Finally, the proposed method is a computational approach and may not be accessible or practical for all healthcare settings. The implementation of the method may require specialized hardware or software, and may not be feasible for smaller clinics or healthcare facilities with limited resources. Despite these limitations, the suggested method indicates an essential stage in melanoma diagnosis and provides a valuable contribution to the expansion of more accurate and efficient recognition implements for this deadly disease.

## 4 Conclusions

At present, cancer as a health issue is a major concern at the world level. Since the timely cancer identification is so effective for on-time cure and recovery of the patients, various approaches has the potential to be utilized for the current goal. Image processing strategies have been defined as non-invasive and simple techniques to detect cancer cells that quicken early diagnosis and finally increment the survival chances of patients. A common kind of cancer is skin cancer which includes about 75 % of all cancers in the world. This study proposed a new wide-ranging technique for the optimum diagnosis of cancer of melanoma from dermoscopy pictures. First, reinforcement learning was used for segmenting the texture of the skin in the input images. Then, a new metaheuristic method is used to categorize and extract attributes. The proposed algorithm was named Enhanced Fish Migration Optimization algorithm which shows good results based on validations. This algorithm was then utilized for feature selection of the extracted attributes from the segmented pictures. Finally, this algorithm was used for the optimal designing of a SVM to categorize the cancerous pictures of support vector machine optimized by the EFMO. The method was finally verified by applying it to the Melanoma dataset of SIIM-ISIC and its accomplishments are compared to different latest algorithms, comprising CNN, Delaunay Triangulation, Fractal analysis, Fusion method, Side-by-Side method, GA, Spotmole, texture Descriptor of MED-NODE, color descriptor of MED-NODE, SVM, ResNet-101 to indicate the efficiency of the suggested technique. Ultimate achievements illustrated the recommended method prepared the finest outcomes for the others. Future research directions for the proposed approach for optimum identification of melanoma cancer could focus on the validation of larger datasets, integration of multiple imaging modalities, incorporation of clinical data, development of real-time diagnostic tools, and conducting clinical trials to establish the clinical utility of the suggested method and diagnose any challenges or boundaries that must be solved.

RETRACTED

## Data availability statement

No data was used for the research described in the article.

## CRediT authorship contribution statement

**Qianqian Liu:** Conceptualization, Data curation, Formal analysis. **Hiroto Kawashima:** Conceptualization, Data curation, Resources, Writing – original draft, Writing – review & editing. **Asad Rezaei sofla:** Data curation, Methodology, Software, Validation, Writing – original draft, Writing – review & editing.

## Declaration of competing interest

The authors declare that they have no known competing financial interests or personal relationships that could have appeared to influence the work reported in this paper.
